The article "Effect of Secreted Frizzled-Related Protein 5 in Mice with Heart Failure" was published in 2022. Journal: Evid Based Complement Alternat Med.

# Effect of Secreted Frizzled-Related Protein 5 in Mice with Heart Failure

**DOI:** 10.1155/2022/1606212

**Published:** 2022-05-31

**Authors:** Pan Hong, Lijie Wang, Hongchao Wang, Min Shi, Bingyan Guo

**Affiliations:** ^1^Department of Cardiology, The Second Hospital of Hebei Medical University, Shijiazhuang 050017, China; ^2^Hebei Key Laboratory of Laboratory Medicine, Shijiazhuang 050017, China

## Abstract

Although some progress has been made in its treatment, heart failure is still one of the most important health problems that endanger public health. This study aims to explore the myocardial protective effect of secreted frizzled-related protein 5 (SFRP5) on mice with heart failure. The mouse model of heart failure was established by using the isoproterenol (ISO) hydrochloride gradient modeling method. The treatment group was injected with 0.02 mg/kg/24 h SFRP5 recombinant protein intraperitoneally 30 minutes after the injection of isoproterenol, and the ISO + phosphate-buffered saline (PBS) group was injected with the same amount of PBS. After intraperitoneal injection of SFRP5 recombinant protein in mice with heart failure, the inflammatory response was reduced, and the left ventricular systolic and diastolic function of heart failure mice and the pathological structure of the myocardial tissue were improved. Compared with the ISO group, the expression level of SFRP5 protein in the ISO + SFRP5 group was increased significantly, the expression levels of Wnt5a and JNK protein were decreased markedly, and the enzyme activities of SOD and GSH-Px in the serum were observably increased, but they were lower than those parameters in the normal group. The SFRP5 recombinant protein has a protective effect on isoproterenol-induced heart failure in mice. The mechanism of action may be related to inhibiting the Wnt5A/JNK signaling pathway and reducing oxidative stress and inflammation. SFRP5 may be one of the therapeutic targets of heart failure.

## 1. Introduction

Heart failure (HF) is a complex clinical syndrome caused by abnormalities in the myocardial structure or function due to various causes. HF has become a global health emergency in the 21^st^ century with extremely high morbidity, disability, and mortality rates. HF is a progressive and irreversible disease, and it is the terminal stage of many cardiovascular diseases. The pathogenesis of HF is related to ventricular remodeling, myocardial fibrosis, inflammation, oxidative stress, and the immune response. At present, there is no cure for HF, and treatment can only delay the gradual deterioration associated with the disease. Secreted frizzled-related protein 5 (SFRP5) is an anti-inflammatory adipocytokine discovered by Ouchi et al. in 2010 that is secreted by white adipose tissues [1]. SFRP5 has anti-inflammatory and metabolic regulatory effects, and it may play an important role in the occurrence and development of cardiovascular diseases.

The article "Effect of Secreted Frizzled-Related Protein 5 in Mice with Heart Failure" was published in 2022. Journal: Evid Based Complement Alternat Med.

SFRP belongs to the secreted glycoprotein family and includes 5 members (SFRP1-5) [2, 3]. The Wnt signaling pathway is involved in the pathophysiological processes of various diseases, such as cell proliferation, differentiation, and apoptosis [4, 5]. The SFRP protein is a secreted Wnt antagonist [6, 7] that can inhibit the activation of the Wnt signaling pathway by binding to Wnt proteins or competitively binding to Fz receptors to regulate the biological functions of cells [8, 9]. SFRP1∼4 can be detected in myocardial tissues in healthy people and in patients with HF. The expression levels of SFRP3 and SFRP4 mRNA in patients with HF were increased. This process may be related to the decrease in *β*-catenin expression and myocardial cell apoptosis [10]. Decreased expression of SFRP1 was detected during the recovery process of patients with HF [11]. As a new anti-inflammatory factor, SFRP1 is a protective factor in the process of heart injury after myocardial infarction. Studies have found that SFRP2 can promote the process of myocardial fibrosis in HF after myocardial infarction. AntiSFRP2 antibody treatment can reduce the process of myocardial fibrosis in HF [12]. SFRP5 can be expressed in hypertrophic cardiomyocytes, and it increases with the increase in cardiomyocyte hypertrophy [13].

As an anti-inflammatory adipokine [1], SFRP5 is involved in cell apoptosis, proliferation, and differentiation. SFRP5 weakens Wnt signaling by binding to Wnt5a, thereby inhibiting the development of cardiovascular diseases such as atherosclerosis [14], coronary heart disease [15, 16], myocardial infarction [17, 18], and myocardial hypertrophy [19]. Nakamura found that SFRP5 may alleviate cardiac inflammation and protect the heart from ischemia/reperfusion injury by inhibiting the WNT5A/JNK signaling pathway [20]. Yu et al. used an exogenous supplementation of the SFRP5 recombinant protein to inhibit the Wnt classical pathway, which could effectively improve renal interstitial fibrosis [21]. The SFRP5 recombinant protein significantly attenuates intrahepatic inflammation and steatosis in the nonalcoholic fatty liver disease by inhibiting the nonclassical pathway, as observed by Lili Chen et al. [22]. Studies have shown that the degree of HF in patients with chronic HF is related to the expression of the SFRP5 protein. However, the protective mechanism of SFRP5 in HF is still unclear, and further research is needed.

The article "Effect of Secreted Frizzled-Related Protein 5 in Mice with Heart Failure" was published in 2022. Journal: Evid Based Complement Alternat Med.

Based on the above elaboration, we hypothesize that SFRP5 is related to the development of HF. In this study, we used isoproterenol (ISO) to establish mouse HF models and exogenously supplemented the SFRP5 recombinant protein to explore the effect of SFRP5 recombinant proteins on the cardiac function and structure of mice with HF and explored its mechanism of action. Our results indicate that SFRP5 is a novel target for the treatment of HF.

## 2. Materials and Methods

### 2.1. Chemical Reagents

Recombinant human SFRP-5 was obtained from R&D Systems (MN, USA). Isoproterenol hydrochloride was purchased from Sigma-Aldrich (St. Louis, MO, USA). Anti-Wnt5A antibody, anti-SFRP5 antibody, anti-IL-1 antibody, anti-IL-6 antibody, and anti-IL-18 antibody were purchased from Abcam (Cambridge, UK). An anti-glyceraldehyde-3 phosphate dehydrogenase (GAPDH) antibody was purchased from Bioworld (MN, USA). Anti-NLRP3 antibody and anti-JNK antibody were purchased from Cell Signaling Technology (Danfoss, MA, USA). Superoxide dismutase (SOD) and glutathione peroxidase (GSH-px) detection kits were purchased from Nanjing Jiancheng Institute of Biological Engineering (Nanjing, China).

### 2.2. Establishment of a Mouse Model of Heart Failure and Experimental Grouping

All animal procedures were in compliance with the approval of the Hebei Medical University (Shijiazhuang, China) Ethics Committee (CNUH IACUC-18023). 5-week-old C57BL/6J male mice of SPF grade were purchased from Beijing Sibeifu Biotechnology Co. Ltd. (Permit Number: SCXK (Jing) 2019-0010). The mice were maintained on a 12-hour light-dark cycle, and they could freely eat and drink for 3 weeks of adaptive feeding. Starting at 8 weeks of age, they were randomly divided into four groups according to their body weight: normal saline (NS) group, ISO group, ISO + PBS group, and ISO + SFRP5 group (*n* = 6). HF was modeled with an isoproterenol hydrochloride gradient: 20 mg/kg on the first day and 5 mg/kg on the 3^rd^ to 14^th^ days to mice with an intraperitoneal injection of isoproterenol. The ISO group, ISO + PBS group, and ISO + SFRP5 group were intraperitoneally injected with isoproterenol according to the above scheme. In the NS group, normal saline was injected subcutaneously once a day for 14 consecutive days. From the day of modeling, the ISO + PBS group was injected with PBS (0.02 mg/kg/24 h) every day, the ISO + SFRP5 group was given SFRP5 recombinant protein (0.02 mg/kg/24 h) every day, and the NS group and ISO group were given the same amount of normal saline for continuous administration for 14 days.

### 2.3. Echocardiography Testing

After 14 days of administration, the chest hair of the mice was shaved with a small animal shaving machine in advance, and the front chest was fully exposed. The mice were anaesthetized by inhalation of isoflurane gas. The mice were fixed on a constant temperature heating plate, the limbs were extended, and the ultrasound lotus mixture was evenly coated on the front chest. The RMV710B ultrasonic probe instrument was chosen in the left ventricular short-axis view, the left ventricular short-axis two-dimensional ultrasound image was saved, and *M* was used to calculate the left ventricular internal systolic diameter (LVIDs), left ventricular internal diastolic diameter (LVIDd), left ventricular rejection fraction (LVEF), and left ventricular fractional shortening (LVFS). At least three measurements were obtained for each mouse, and the average value of 3 cardiac cycles was recorded.

The article "Effect of Secreted Frizzled-Related Protein 5 in Mice with Heart Failure" was published in 2022. Journal: Evid Based Complement Alternat Med.

### 2.4. Assessment of the Indices of the Heart Weight

After measuring the heart function, the mice were sacrificed by cervical dislocation, the thoracic cavity was opened to expose the heart, the heart was quickly removed, and the heart tissue was fully washed with normal saline. The water was dried with a filter paper, and the heart was weighed (mg). The calculation of the heart mass index (HMI) is as follows: heart mass index (HMI) = heart weight (mg)/mouse weight (g).

### 2.5. Myocardial Histopathology

The left ventricle sections were collected, fixed with 4% paraformaldehyde, and embedded in paraffin. The tissues were sectioned in conventional paraffin and stained with hematoxylin and eosin (HE). The sections were inspected by an experienced observer using an optical microscope (OLYMPUS, Japan) who was blinded to the treatment plan. The pathological structure of the myocardial tissue of each group of mice was observed.

### 2.6. Western Blotting

Total protein was extracted from cardiomyocytes. According to the results of protein quantification, 20 micrograms of total protein sample and 5× protein gel electrophoresis loading buffer were added, mixed gently, denatured at 95°C for 10 minutes, and immediately placed on ice for use. The protein sample was gently added to the gel well, the electrophoresis apparatus was set to a voltage-stabilized state, the power supply was turned on, and the voltage was adjusted to 80 V to pass the sample through the concentrated gel and separation gel (the voltage was approximately 8 V/cm). Once the electrophoresis brought the dye to the proper position of the separation gel, the electrophoresis was stopped. After the gel electrophoresis was completed, the protein bands separated on the gel were transferred to a solid support by transfer electrophoresis, and the primary antibody was diluted with a blocking solution. The blocked membrane was placed directly into the working solution of the primary antibody and reacted overnight at 4°C. The washed primary antibody reaction membrane was placed into the secondary antibody working solution (1 : 10,000) and incubated for 1 hour. Universal developer powder and acid fixing powder (Tianjin Tianluhai Photosensitive Material Factory) were used to visualize the protein strips. ImageJ software was used to analyze the gray value. The ratio of the detected protein band density to the GAPDH protein band density was used for statistical analysis.

The article "Effect of Secreted Frizzled-Related Protein 5 in Mice with Heart Failure" was published in 2022. Journal: Evid Based Complement Alternat Med.

### 2.7. Oxidative Stress Marker Detection

After the test, the eyeballs of the mice were removed, and the blood was placed in an anticoagulation tube, agglomerated at room temperature for 1 hour, and centrifuged at 3000 r/min for 15 minutes. The supernatant was aspirated into a clean Eppendorf (EP) tube and stored at −80°C for later use. The serum SOD and GSH-Px activities were determined according to the kit instructions.

### 2.8. Statistical Analyses

SPSS 20.0 software was used for statistical analysis. All data are expressed as the mean ± standard deviation (SD). One-way analysis of variance (ANOVA) and Student–Newman–Keuls' test were used to make pairwise comparisons between groups. *P* < 0.05 was considered statistically significant.

## 3. Results

### 3.1. SFRP5 Recombinant Protein Reduces the Cardiac Hypertrophy in Mice Caused by Isoproterenol

As shown in Figure 1, mouse hearts showed marked hypertrophy in the ISO group and the ISO + PBS group. However, treatment with recombinant SFRP5 protein attenuated isoproterenol-induced cardiac hypertrophy. Compared with that in the NS group, the ratio of heart weight to body weight (HW/BW) increased significantly. Compared with that in the ISO group, the HW/BW of the ISO + SFRP5 group was observably lower.

### 3.2. SFRP5 Recombinant Protein Improves the Left Ventricular Dysfunction in Mice with Heart Failure

Fourteen days after the model was created, according to the analysis of the measured and calculated values of cardiac ultrasound in each group, the LVEDs and LVEDd of the heart of the ISO group were markedly increased compared with the LVEDs and LVEDd of the hearts of the NS group, and the LEVF and FS were significantly decreased. Changes in these parameters indicate that isoproterenol can cause an impaired cardiac function in mice. After intraperitoneal injection of the SFRP5 recombinant protein, the LEVF and FS values of mouse hearts were higher than the LEVF and FS values of mouse hearts in the ISO and ISO + PBS groups; the LVEDd value was decreased (*P* < 0.05), and ventricular contraction and diastolic function were markedly improved (Figure 2). The test results showed that the SFRP5 recombinant protein can improve myocardial contractile and diastolic function after HF.

The article "Effect of Secreted Frizzled-Related Protein 5 in Mice with Heart Failure" was published in 2022. Journal: Evid Based Complement Alternat Med.

### 3.3. SFRP5 Recombinant Protein Reduces the Levels of Inflammatory Factors in the Myocardial Tissue of Mice with Heart Failure

The changes in inflammatory factors in the myocardium of each group of mice were detected by western blotting (Figure 3). The results showed that compared with the NS group, the expression of NLRP3 protein and other inflammatory factors, such as IL-1*β*, IL-6, and IL-18, in the myocardial tissue of the ISO group and ISO + PBS group increased significantly (*P* < 0.01). After intervention with the SFRP5 recombinant protein, the expression of the abovementioned inflammatory factors in the myocardium of the ISO + SFRP5 group mice decreased observably, and the difference was statistically significant (*P* < 0.05).

### 3.4. SFRP5 Recombinant Protein Reduces Serum Oxidative Stress Levels in Heart Failure

The SOD and GSH-Px levels in mouse serum were measured. After intraperitoneal injection of ISO, the levels of SOD and GSH-Px in the serum of mice were significantly reduced. Compared with the ISO group, the ISO + SFRP5 group mice had markedly enhanced SOD and GSH-Px activities in the serum, and the difference was statistically significant (*P* < 0.05). The results showed that the SFRP5 recombinant protein can markedly enhance the levels of SOD and GSH-px in the serum of mice with HF induced by ISO (Figure 4).

### 3.5. SFRP5 Recombinant Protein Improves the Myocardial Tissue Pathological Structure in Mice with Heart Failure

Histological examination showed that the cardiomyocytes of the NS group were arranged neatly, and the shapes were relatively regular. After the injection of ISO, the mouse cardiomyocytes were disordered, and inflammatory cells had infiltrated. A large number of vacuoles, severe distortion, and deformation could be seen, and collagen fiber deposition between the myocardial tissues was obviously proliferated. After the injection of the SFRP5 recombinant protein, the degree of injury and scope of the mouse myocardial cells were significantly reduced (Figure 5).

### 3.6. SFRP5 Recombinant Protein Inhibits Wnt5A/JNK Signaling Pathway Activation

To verify whether SFRP5 recombinant protein can inhibit the activation of the Wnt5A/JNK signaling pathway, thereby protecting ISO-induced HF mice, we used western blotting to detect the expression of related proteins. Compared with mice in the NS group, the expression of SFRP5 in the myocardial tissue of the mice was significantly decreased after ISO injection, and the expression of WNT5A and JNK was observably increased. In contrast to levels in the mice in the ISO group and the ISO + PBS group, exogenous supplementation with the SFRP5 recombinant protein upregulated the expression of SFRP5 in myocardial tissues, which inhibited the WNT5A/JNK signaling pathway and ultimately alleviated ISO-induced HF in mice (Figure 6).

The article "Effect of Secreted Frizzled-Related Protein 5 in Mice with Heart Failure" was published in 2022. Journal: Evid Based Complement Alternat Med.

## 4. Discussion

In this study, we determined that SFRP5 is a protective factor for HF. The mechanism can be attributed to the regulation of the Wnt5A/JNK signaling pathway.

Isoproterenol can induce myocardial cell damage, necrosis, oxidative stress, and cardiac metabolism changes; enhance myocardial contractility; and simulate pressure-overloaded HF. ISO has the advantages of noninvasiveness, high safety, and good uniformity and is widely used in current animal models of HF [23, 24].

Pathologic cardiac hypertrophy is the most important pathophysiological basis leading to HF. SFRP5 has been shown to be expressed in cardiomyocytes, and SFRP5 is upregulated in cardiomyocyte hypertrophy and plays a key role in reversing the progression of cardiac hypertrophy and cardiomyopathy through the AT1-R/Rho/ROCK 1/JNK signaling pathway. Our research results showed that after the injection of ISO-induced HF in mice, the myocardium of the mice was severely damaged, and myocardial hypertrophy was observed. In contrast, after intervention with the SFRP5 recombinant protein, the weight of the mouse hearts was decreased significantly, indicating that the SFRP5 recombinant protein can reverse ISO-induced cardiac hypertrophy. Consistent with the assessment of myocardial hypertrophy, HE staining clearly showed that the pathological structure of myocardial tissues in the ISO group was disordered, and collagen deposition was increased. However, SFRP5 treatment visibly reduced collagen deposition in the heart and reduced myocardial damage.

Clinical studies have found that with increasing cardiac function grade, the LV ejection fraction level decreased, the left ventricular end-diastolic diameter increased, and there was a compensatory increase in the SFRP5 expression. To evaluate the effect of SFRP5 on mice with HF, this study included hemodynamic parameters. Isoproterenol-treated mice showed obvious cardiac dysfunction, LVEDs and LVEDd values distinctly increased, and LEVF and FS values clearly decreased. After treatment with SFRP5 recombinant protein, the systolic and diastolic functions of the mouse hearts were significantly improved.

Studies have shown that inflammation and oxidative stress are involved in the formation of HF [19]. During the pathogenic process of HF, cardiomyocytes secrete large amounts of inflammatory factors, leading to oxidative stress damage in cardiomyocytes, which can contribute to the pathological remodeling of myocardial and cardiovascular diseases and promote the progression of HF. SFRP5 can not only enhance adipocyte hypertrophy by inhibiting oxidative metabolism but can also act as an anti-inflammatory adipokine that is widely involved in apoptosis, proliferation, and differentiation and is capable of exerting anti-inflammatory as well as metabolic regulatory roles by attenuating Wnt signaling by binding to Wnt5a. Therefore, we detected the expression levels of inflammatory factors in the myocardial tissue of mice and used a kit to detect the levels of SOD and GSH-Px in the serum of mice. The levels of SOD and GSH-Px in the serum of mice in the ISO group were evidently reduced, while the expression of inflammatory factors in myocardial tissue was obviously increased. After intervention with the SFRP5 recombinant protein, the abovementioned abnormalities were significantly restored, indicating that the SFRP5 recombinant protein can inhibit oxidative stress and inflammatory reactions, improve myocardial damage, and exert a protective role against isoproterenol-induced myocardial damage.

The article "Effect of Secreted Frizzled-Related Protein 5 in Mice with Heart Failure" was published in 2022. Journal: Evid Based Complement Alternat Med.

A large amount of evidence show that the Wnt signaling pathway is closely related to cardiovascular diseases [13]. The processes of cardiomyocyte proliferation, differentiation, and apoptosis [25, 26]; cardiac remodeling; and HF are all accompanied by the participation of Wnt-Fzd signaling pathway molecules. The Wnt signaling pathway is likely to become a new target for prevention and treatment [22, 27]. SFRPs can inhibit the activation of the Wnt signaling pathway by binding to Wnt proteins or competitively to Fz receptors and can regulate the biological function of cells. As a member of the SFRP family, SFRP5 plays a protective role in disease processes, such as atherosclerosis, and has metabolic relevance. In this study, western blotting was used to detect the expression levels of Wnt5A and JNK proteins in mouse myocardial tissues. After the injection of isoproterenol, the expression levels of Wnt5A and JNK proteins in myocardial tissues were significantly increased. After treatment with SFRP5 recombinant protein, the Wnt5A and JNK protein expression was recovered.

There are also some limitations to our study. ISO-induced mouse models are currently widely used to mimic advanced HF. Our experiments in mice could not rule out the possible contribution of other metabolites to the protection against ISO-induced HF. Moreover, in vitro experiments are needed to further explore the protective mechanisms of SFRP5. Additionally, the experimental sample size was small, and experimental error may be present. Finally, investigation of the progressive dynamics of the observation indicators was lacking. Therefore, the experimental accuracy may be affected.

The article "Effect of Secreted Frizzled-Related Protein 5 in Mice with Heart Failure" was published in 2022. Journal: Evid Based Complement Alternat Med.

## 5. Conclusion

The SFRP5 recombinant protein can improve HF in mice caused by isoproterenol. The mechanism may be related to inhibiting the activation of the Wnt5A signaling pathway and reducing oxidative stress and inflammation. Our study may provide new strategies and ideas for the clinical prevention and treatment of HF.

## Figures and Tables

**Figure 1:** Effect of SFRP5 recombinant protein on myocardial hypertrophy and the heart weight index in isoproterenol-induced myocardial hypertrophy and HF mice. After treatment termination, the mice were euthanized, and HW and BW were measured. (a) Representative hearts of mice in each of the four groups and (b) heart weight index (*n* = 6). ^*∗∗*^*P* < 0.01 compared with the NS group. ^##^*P* < 0.01 compared with the ISO group.

**Figure 2:** Effect of the SFRP5 recombinant protein on UCG changes in ISO-induced HF in mice. (a) Representative M-mode echocardiograms of mice in the four groups. (b) Comparison of the cardiac function in the four groups of mice (*X* ± *S*). Each value represents the mean of 6 experiments ± SEM (*n* = 6). ^*∗∗*^*P* < 0.01 compared with the NS group. ^#^*P* < 0.05, ^##^*P* < 0.01 compared with the ISO group.

**Figure 3:** Effect of SFRP5 recombinant protein on the expression of myocardial tissue inflammatory factors in the four groups of mice. ^*∗∗*^*P* < 0.01 compared with the NS group. ^#^*P* < 0.05, ^##^*P* < 0.01 compared with the ISO group.

**Figure 4:** Comparison of the serum oxidative stress levels in the four groups of mice. At the end of the experiment, mouse blood was collected. The mouse serum SOD and GSH-Px expression levels were measured using a kit. ^*∗∗*^*P* < 0.01 compared with the NS group. ^##^*P* < 0.01 compared with the ISO group.

**Figure 5:** Effects of recombinant SFRP-5 proteins on the pathological structure of the myocardium in ISO-induced HF in mice. The NS group (a) showed the normal histological structure of the cardiac muscle. The ISO group (b) and ISO + PBS group (c) showed severe cardiac insult, marked inflammatory cell infiltration, and edema between muscle fibers. The ISO + SFRP5 group (d) demonstrated almost normal cardiac muscles.

**Figure 6:** Protein expression of SFRP5, Wnt5A, and JNK in the four groups of mice. Heart samples were collected after administration. Equal amounts of sample were subjected to western blotting, as described in the Materials and Methods.  ^*∗*^ ^*∗*^*P* < 0.01 compared with the NS group. ^##^*P* < 0.01 compared with the ISO group.

## Data Availability

No data were used to support the findings of the study.
